The article "Clinical Feature-Based Machine Learning Model for 1-Year Mortality Risk Prediction of ST-Segment Elevation Myocardial Infarction in Patients with Hyperuricemia: A Retrospective Study" was published in 2021. Journal: Comput Math Methods Med.

# Clinical Feature-Based Machine Learning Model for 1-Year Mortality Risk Prediction of ST-Segment Elevation Myocardial Infarction in Patients with Hyperuricemia: A Retrospective Study

**DOI:** 10.1155/2021/7252280

**Published:** 2021-07-05

**Authors:** Zhixun Bai, Jing Lu, Ting Li, Yi Ma, Zhijiang Liu, Ranzun Zhao, Zhenglong Wang, Bei Shi

**Affiliations:** ^1^Program of Artificial Intelligence in Medicine, College of Medicine, Soochow University, Suzhou 215123, China; ^2^Department of Internal Medicine, The Second Affiliated Hospital of Zunyi Medical University, Zunyi 563000, China; ^3^Department of Cardiology, Affiliated Hospital of Zunyi Medical University, Zunyi, China; ^4^Department of Pathology, Zunyi Medical and Pharmaceutical College, Zunyi 563006, China

## Abstract

Accurate risk assessment of high-risk patients is essential in clinical practice. However, there is no practical method to predict or monitor the prognosis of patients with ST-segment elevation myocardial infarction (STEMI) complicated by hyperuricemia. We aimed to evaluate the performance of different machine learning models for the prediction of 1-year mortality in STEMI patients with hyperuricemia. We compared five machine learning models (logistic regression, *k*-nearest neighbor, CatBoost, random forest, and XGBoost) with the traditional global (GRACE) risk score for acute coronary event registrations. We registered patients aged >18 years diagnosed with STEMI and hyperuricemia at the Affiliated Hospital of Zunyi Medical University between January 2016 and January 2020. Overall, 656 patients were enrolled (average age, 62.5 ± 13.6 years; 83.6%, male). All patients underwent emergency percutaneous coronary intervention. We evaluated the performance of five machine learning classifiers and the GRACE risk model in predicting 1-year mortality. The area under the curve (AUC) of the six models, including the GRACE risk model, ranged from 0.75 to 0.88. Among all the models, CatBoost had the highest predictive accuracy (0.89), AUC (0.87), precision (0.84), and F1 value (0.44). After hybrid sampling technique optimization, CatBoost had the highest accuracy (0.96), AUC (0.99), precision (0.95), and F1 value (0.97). Machine learning algorithms, especially the CatBoost model, can accurately predict the mortality associated with STEMI complicated by hyperuricemia after a 1-year follow-up.

## 1. Introduction

The most common cardiovascular diseases currently include hypertension, heart failure, coronary atherosclerosis, and myocardial infarction (MI); there is widespread interest in these conditions, as they are associated with high morbidity and mortality. In recent years, the incidence and death rate associated with MI have increased in China. The incidence of MI, though not strongly associated with the regions in China, has been found to increase with age [1]. Research has shown that MI typically starts to develop in young and middle-aged people. Therefore, the prevention, detection, and treatment of MI have become an area of interest among medical experts and scholars. In recent years, uric acid (UA) has been increasingly recognized as a well-known cardiovascular risk factor, along with hypertension, diabetes, chronic kidney disease (CKD), and obesity [2–7]. Although it is unclear whether UA is an independent predictor of cardiovascular disease, recent retrospective studies have demonstrated that hyperuricemia is an independent predictor of short- and long-term mortality in patients with AMI [8–10]. Machine learning is a multidisciplinary field involving artificial intelligence, computational complexity theory, probability and statistics, cybernetics, information theory, philosophy, physiology, neurobiology, and other disciplines that can be characterized by system self-improvement. Machine learning was developed from the research method based on neuron models and function approximation theory; rule learning and decision tree learning were then incorporated based on symbolic calculus [11]. Furthermore, machine learning plays an essential role in clinical practice and cardiology. Each machine learning algorithm has its advantages in different fields. Previous studies have found that machine learning has good predictive power in predicting intrahospital mortality and short-term prognosis in acute MI. However, imbalanced data distribution and quality of deaths and survivors, that may lead to misclassification, are great challenges in machine learning. If the model evaluation places excessive emphasis on the area under the curve (AUC) index, it may ignore the weakness of truly predicting actual deaths. At present, there has been no research for developing a more comprehensive machine learning prediction model for the prognosis of ST-segment elevation myocardial infarction (STEMI) patients with hyperuricemia. Therefore, in this study, we evaluated multiple performance indicators for predicting 1-year mortality in STEMI patients with hyperuricemia, by using different machine learning models including logistic regression (LR), *k*-nearest neighbor (KNN), CatBoost, random forest (RF), and XGBoost. We then compared these models with the traditional GRACE risk score. To improve the prediction accuracy of imbalanced learning, we used SMOTEENN, a hybrid sampling algorithm of synthetic minority oversampling technique (SMOTE), and edited nearest neighbor (ENN) algorithms to oversample the minority class by creating synthetic samples.

The article "Clinical Feature-Based Machine Learning Model for 1-Year Mortality Risk Prediction of ST-Segment Elevation Myocardial Infarction in Patients with Hyperuricemia: A Retrospective Study" was published in 2021. Journal: Comput Math Methods Med.

## 2. Materials and Methods

### 2.1. Patients

This investigation followed the Transparent Reporting of a Multivariable Prediction Model for Individual Prognosis or Diagnosis (TRIPOD) reporting guidelines for cohort studies [12]. We enrolled consecutive patients aged >18 years diagnosed with STEMI at the Affiliated Hospital of Zunyi Medical University between January 2016 to January 2020 (Figure 1). The inclusion criteria were as follows: (1) increase or occurrence of ischemic chest discomfort at rest; (2) elevation of ST − segment ≥ 0.1 mV; (3) elevation of ST-segment in two consecutive leads; (4) elevated cardiac troponin I (≥0.03 *μ*g/L) or cardiac troponin T levels (≥42 ng/L); (5) diagnosed with hyperuricemia on admission; (6) no history of recent nephrotoxic drug intake; and (7) receipt of emergency percutaneous coronary intervention (PCI) treatment. The use of drugs was based on the treatment standards recommended by the published guidelines. Research approval was obtained from the Ethics Committee of the Affiliated Hospital of Zunyi Medical University (approval No. KLL [2020]0144). The need for written informed consent was waived owing to the retrospective nature of the study.

### 2.2. Outcomes

The primary outcome was defined as cardiac and sudden deaths during the 1-year clinical follow-up after discharge. Patients who had died during hospital admission were excluded from the analysis; the follow-up period ended in January 2021. All eligible patients enrolled in this study were followed up through telephone interviews or outpatient visits.

### 2.3. Candidate Predictors

Data on demographic characteristics, disease, electrocardiographic findings, laboratory parameters on admission, and in-hospital events were obtained from the patient's medical records. Data on baseline characteristics, demographics (age and gender), risk factors (hypertension, diabetes, current smoking, family history), nonweekday admission (NWDS), delay (defined as patient FMC > 12 hours), medical history (previous stroke, previous CKD), and electrocardiography (ECG) findings (inferior, anterior, right ventricular, and other) were all obtained from our electronic database. Hyperuricemia was defined by serum UA levels of >7 mg/dL (417 mmol/L) in men and >6 mg/dL (357 mmol/L) in women at admission. The patient data collected included demographic information, baseline characteristics at admission, diagnosis and treatment during hospitalization, diseased vessel identified during procedure, diagnosis at discharge and drug treatment, and comorbidities, such as hypertension, diabetes, and renal disease; in total, 41 characteristics were analyzed. Based on TRIPOD reporting guidelines, the rule of thumb for sample size is to have at least 10 outcome events per variable (EPV).

The article "Clinical Feature-Based Machine Learning Model for 1-Year Mortality Risk Prediction of ST-Segment Elevation Myocardial Infarction in Patients with Hyperuricemia: A Retrospective Study" was published in 2021. Journal: Comput Math Methods Med.

### 2.4. Data Collection

In our data source, all attributes that can be subdivided are categorized into independent classes, and each class generates a new attribute. The new attribute is encoded with the one-hot encoding rule. The data were susceptible to incorrect notation by the researcher; data cleansing and editing, consisting of removing typographical errors, and reviewing data quality in data reporting, were performed by a second researcher to avoid a flawed model training process. Assessment of predictors in our study has been performed without knowledge of the participant's outcome. A single investigator assessed all demographic information and clinical data and was blinded to the outcome of mortality. Additionally, a different researcher assessed the plausibility of the results regarding the outcome of mortality.

### 2.5. Missing Values

Complete case data were collected from the electronic health records (EHRs) and analyzed; all variables can be queried in the EHRs. Some patients were excluded as they refused to undergo the candidate predictor laboratory test or failed to comply with 1-year follow-up.

### 2.6. Statistical Analysis

Continuous variables are presented as the mean ± standard deviation, and classified variables are indicated by counts and percentages. Differences in baseline characteristics between groups were analyzed using the independent sample *t*-test. The Mann–Whitney *U* test was used for continuous variables, and the chi-square test or Fisher's exact test was used for categorical variables. The previously described GRACE risk score was used to analyze mortality, and it was calculated according to the published formula [13]. Five machine learning classifiers (LR, KNN, CatBoost, RF, and XGBoost) and the ensemble model were used as the supervised machine learning methods to predict survival status after 1-year follow-up. In order to solve the problem of imbalanced data classification owing to medical diagnosis, we used SMOTEENN, a hybrid sampling algorithm of SMOTE and ENN algorithms; this helped to oversample the minority (death cases) class by creating synthetic samples, followed by cleaning the mislabeled instances. Supervised learning aims to establish a concise model of outcome type distribution (called label in machine learning), based on predictor parameters [14]. All models were validated by 10-fold crossvalidation. In feature engineering, all classification features were transformed by one-hot encoding, and the missing values were provided by the missForest method. Compared with the traditional chain multifilling method, this method results in significant performance improvement [14–16]. The following indicators were used to define model performance: AUC, recall, precision, and F1 value. Python (version 3.7, https://www.python.org/) was used for all statistical analyses.

The article "Clinical Feature-Based Machine Learning Model for 1-Year Mortality Risk Prediction of ST-Segment Elevation Myocardial Infarction in Patients with Hyperuricemia: A Retrospective Study" was published in 2021. Journal: Comput Math Methods Med.

## 3. Results and Discussion

Between January 2016 and January 2020, a total of 738 STEMI patients registered in the database met the inclusion criteria. After excluding those who were lost to follow-up (*n* = 82), 656 patients were enrolled in this study. The patients' average age was 62.5 years (±13.6 years), and 83.6% were male. All patients underwent emergency PCI. The median follow-up duration was 25 months, and 91 patients died within 1 year of admission, resulting in a mortality rate of 13.8%.  Table 1 summarizes the differences in demographic information, admission baseline characteristics, and diseased vessels between the patients who survived and those who died. Considering the imbalance of classification data among samples (death cases : survival cases = 91 : 565), five machine learning algorithms (logistic regression, KNN, RF, XGBoost, and CatBoost) were developed to predict the 1-year mortality rate with all available features. RF (accuracy = 0.89, AUC = 0.88) and CatBoost (accuracy = 0.89, AUC = 0.87) provided similar AUC values in our study, and the predicted performance was higher than that of the traditional GRACE score. As a traditional risk assessment tool, GRACE (accuracy = 0.84, AUC = 0.80) also showed good discriminatory ability in our study (Table 2). The RF classifier outperformed the other models in terms of the AUC crossvalidation results (Figure 2). This study used SMOTEENN to further optimize the models; thus, the performance of all machine learning models was improved significantly (Table 2, Figure 3). After using SMOTEENN to generate more minority class samples, the CatBoost model (accuracy = 0.96, AUC = 0.99, recall = 0.98, precision = 0.95, F1 value = 0.97) demonstrated the highest performance (Figure 4). We investigated the possibility of combining different models to improve performance. In particular, we tried several ensembles and combination methods, including training of the above classifiers and combining their predictions to check whether combination is better than any single classifier (Table 3). The CatBoost was separately integrated with Bagging and Boosting. Further, when the prediction probability of each model was used as the combination rule through the combination of LR, KNN, and XGBoost models after 10-fold crossvalidation, the performance of some models partially improved (recall from 0.33 to 0.53; F1 value from 0.44 to 0.58) compared with that of a single model. This shows that different models can be regarded as partially complementary. When the other abovementioned models were included in the integration method according to different combinations, very similar results were obtained.

The article "Clinical Feature-Based Machine Learning Model for 1-Year Mortality Risk Prediction of ST-Segment Elevation Myocardial Infarction in Patients with Hyperuricemia: A Retrospective Study" was published in 2021. Journal: Comput Math Methods Med.

Owing to the recent widespread development of chest pain centers in China, 70.8% of patients with acute STEMI were admitted to the hospital within 12 hours of onset and received prompt reperfusion treatment. Hospital mortality rates have therefore decreased significantly. Timely and effective revascularization treatment is key for the reduction of mortality and improved prognosis following AMI. The rescue system based on chest pain centers has played an essential role in improving the timeliness of revascularization in AMI patients and in reducing mortality.

Previous studies have confirmed that baseline renal dysfunction and acute kidney injury are strong predictors of in-hospital and long-term adverse cardiovascular outcomes after STEMI complicated by cardiogenic shock [17]. STEMI-related mortality is considerably higher in those who have had unsuccessful invasive procedures or those with diabetes, chronic kidney failure, or high serum lactate or glucose levels [17, 18].

UA is the final product of purine metabolism and is metabolized by xanthine oxidase. Hyperuricemia can lead to gout and nephrolithiasis; it has also been implicated as an indicator for diseases, such as the metabolic syndrome, diabetes mellitus, cardiovascular disease, and chronic renal disease. Previous studies have suggested that hyperuricemia with STEMI is associated with a poor prognosis and a high incidence of death and major adverse cardiovascular events (MACEs) [19]. Although the pathophysiological mechanisms of adverse reactions to hyperuricemia have not been fully elucidated, it appears to be multifactorial. In the light of the experimental evidence, hyperuricemia was linked to a variety of proatherogenic processes, including increased oxidative stress, inhibition of endothelial nitric oxide, activation of the renin-angiotensin system, and increase in the microvascular damage via endothelial dysfunction and vascular smooth muscle cell proliferation [20–23].

There is currently no effective evaluation method to predict the long-term prognosis of these patients. GRACE risk scores can be used to estimate follow-up results after acute coronary syndrome. Although Asian populations were not included during the development of the model, the use of GRACE revealed a good discriminatory accuracy in predicting both short-term and long-term MACEs in Asian patients with MI [24]. Our cohort had a median follow-up duration of 25 months, similar to those of previously published studies (accuracy = 0.84, AUC = 0.8). However, the statistical methods in these traditional assessment tools include the Cox proportional hazard regression model. Researchers make presumptions and employ subjective feature selection before model fitting, potentially leading to loss of information [15]. As we enter the era of precision medicine, the demand for risk assessment tools has gained importance. In cases where the research goal is to generate a model that can predict the results most accurately, machine learning algorithms may be more advantageous compared to traditional regression methods. First, machine learning methods can compute multiple related predictions, nonlinear relationships, and the internal interaction between predictors and end events in large datasets. Second, as a critical component of the TRIPOD original declaration report [25], the model should be verified after establishment. In cases where the machine learning method is used, model performance is more robust after external verification. In this study, we compared several standard machine learning methods and performed 10-fold crossinternal verification of the dataset in the absence of external data to ensure model robustness. However, in the traditional regression model, internal validation is not necessary, because one (ideally) posits an analytic model before fitting it to the data [15]. Considering the different effects of each machine learning method in solving medical professional problems, this study compares the efficiency and robustness of various machine learning methods with that of the traditional risk score to obtain more cautious results.

The article "Clinical Feature-Based Machine Learning Model for 1-Year Mortality Risk Prediction of ST-Segment Elevation Myocardial Infarction in Patients with Hyperuricemia: A Retrospective Study" was published in 2021. Journal: Comput Math Methods Med.

In previous studies, machine learning methods showed a better ability to predict short-term mortality after STEMI, while XGBoost showed better predictive ability than other machine learning models in patients with anterior wall STEMI [14]. Gradient boosted tree (GBT) methods, such as XGBoost, RF, and CatBoost, provided similar AUC values in our study. However, after model optimization, the CatBoost model showed more accurate prediction ability. The CatBoost algorithm, which was released in 2017, LightGBM, and XGBoost are the three mainstream machine learning methods for GBT. The CatBoost algorithm is a GBT framework based on an asymmetrical decision tree (oblivious trees) algorithm, with only a few parameters; it supports class variables and has high accuracy. It mainly addresses the issue of dealing with category features efficiently and reasonably.

Furthermore, to improve the algorithm's accuracy and generalization ability, a new method was proposed to account for gradient deviation (gradient bias) and prediction partial (prediction shift) problems. As a new algorithm released in 2017, this method can account for category features in clinical practice and can effectively prevent overfitting; its high training accuracy has provoked widespread interest. Our study also demonstrated the high accuracy of the model. Interestingly, under the premise of the imbalance of clinical samples, the machine learning method with the oversampling technique SMOTEENN could significantly improve performance. SMOTEENN is a hybrid sampling technique of SMOTE and ENN algorithms, that is often employed to oversample the minority class by creating synthetic samples, followed by cleaning of mislabeled instances [26]. It is essential to be aware of the dramatic effects of these synthetic sampling techniques on machine learning models.

The article "Clinical Feature-Based Machine Learning Model for 1-Year Mortality Risk Prediction of ST-Segment Elevation Myocardial Infarction in Patients with Hyperuricemia: A Retrospective Study" was published in 2021. Journal: Comput Math Methods Med.

Our research has several limitations. Owing to the retrospective design of this study, the process of patient data collection may have been accompanied by a risk of bias. Further, this was a single-center study, including only Chinese patients. Under the premise of the imbalance of clinical samples, the machine learning method based on clinical data alone could not obtain a higher AUC value; even the oversampling technique could not significantly improve performance. Second, although the machine model based on hybrid sampling technology has achieved excellent performance in this study, the samples in hybrid sampling technology are computer-generated samples and not real patients; thus, making a more accurate assessment of the prognosis of STEMI patients with hyperuricemia using big clinical data requires further analysis using a more extensive dataset. Despite the abovementioned limitations, our study also has some strengths. The results provide an effective and robust method for predicting 1-year mortality in patients with STEMI complicated by hyperuricemia, through the crossvalidation of machine learning models. Further study requires the combination of social factors, environmental parameters, and phenotypic information (such as genome or proteomics data) in MI for prognostic prediction.

## 4. Conclusion

In conclusion, the predictive ability of machine learning methods is significantly higher than that of the traditional statistical scoring model. The machine learning model will be helpful for the prediction and early detection of MACEs in patients with STEMI complicated by hyperuricemia. In addition, in cases of clinically unbalanced samples, the oversampling technology can significantly improve model performance and ability; however, it is essential to be aware of the dramatic effects of the synthetic sampling techniques on models. There is still uncharted territory in clinical medicine, and methods for accurately predicting the occurrence of some diseases or adverse events will remain the enduring focus of clinical research. Although machine learning presently appears to have good predictive effect, further reasonable and scientific verification is required.

The article "Clinical Feature-Based Machine Learning Model for 1-Year Mortality Risk Prediction of ST-Segment Elevation Myocardial Infarction in Patients with Hyperuricemia: A Retrospective Study" was published in 2021. Journal: Comput Math Methods Med.

## Figures and Tables

**Figure 1:** A flow diagram showing the study process.

**Figure 2:** ROC analysis result of five classifiers and GRACE for the prediction of 1-year mortality with all available features.

**Figure 3:** ROC analysis result of five classifiers with SMOTEENN.

**Figure 4:** CatBoost model performance visualization. (a) ROC curve. (b) Precision-recall curve. (c) Confusion matrix. (d) Classification report. (e) Feature importance. (f) Decision boundary.

**Table 1:** Comparison of characteristics of patients with and without mortality in the cohort.

Variables	Total (*n* = 656)	Survival (*n* = 565)	Death (*n* = 91)	*P* value
Demographic characteristics				
Sex, *n* (%)				0.008
Female	107 (16)	83 (15)	24 (26)	
Male	549 (84)	482 (85)	67 (74)	
Age, y	64.00 (52, 74)	63.00 (51, 73)	70.00 (59, 78)	<0.001
Smoking, *n* (%)	453 (69)	396 (70)	57 (63)	0.192
Weekend on admission, *n* (%)	248 (38)	205 (36)	43 (47)	0.059
Delay, *n* (%)	167 (25)	133 (24)	34 (37)	0.007
Vascular risk factors				
Hypertension, *n* (%)	380 (58)	326 (58)	54 (59)	0.857
Diabetes mellitus, *n* (%)	121 (18)	98 (17)	23 (25)	0.096
Prior-stroke, *n* (%)	35 (5)	30 (5)	5 (5)	1
CKD, *n* (%)	152 (23)	122 (22)	30 (33)	0.024
Clinical data				
HR, beats/min	80 (72, 92)	80.00 (72, 91)	85 (73, 106)	0.003
SBP, mmHg	124 (108, 140)	127 (110, 143)	111 (92, 129)	<0.001
DBP, mmHg	80 (68, 91)	80 (70, 92)	74 (58, 85)	<0.001
Shock_index	0.65 (0.55, 0.77)	0.64 (0.54, 0.75)	0.75 (0.61, 1.04)	<0.001
Electrocardiographic data				
Inferior, *n* (%)	300 (46)	263 (47)	37 (41)	0.351
Anterior, *n* (%)	322 (49)	276 (49)	46 (51)	0.851
Other, *n* (%)	21 (3)	16 (3)	5 (5)	0.194
Right ventricular, *n* (%)	7 (1)	6 (1)	1 (1)	1
Laboratory examinations on admission				
WBC, ^∗^10^9^/L	11.27 (8.60, 14.19)	10.97 (8.34, 13.57)	13.92 (10.56, 19.51)	<0.001
Neutrophil count, ^∗^10^9^/L	8.85 (6.34, 11.83)	8.46 (6.11, 11.19)	11.40 (8.43, 16.26)	<0.001
NLR	6.65 (3.89, 10.77)	6.25 (3.78, 9.85)	9.74 (5.89, 14.93)	<0.001
PLR	149.03 (104.31, 224.60)	148.96 (107.43, 220.27)	151.40 (81.96, 250.07)	0.518
MLR	0.54 (0.37, 0.82)	0.51 (0.36, 0.76)	0.75 (0.41, 1.12)	<0.001
SIRI	4.51 (2.63, 8.44)	4.19 (2.47, 7.39)	8.41 (4.38, 15.27)	<0.001
SII	1285.43 (746.84, 2247.28)	1233.05 (735.30, 2139.17)	1923.99 (894.50, 2898.80)	0.003
HB, g/L	139.00 (123.00, 154.00)	140.00 (124.00, 155.00)	128.00 (115.00, 147.00)	0.001
RBC, ^∗^10^12^/L	4.54 (3.98, 5.01)	4.58 (4.05, 5.02)	4.21 (3.71, 4.88)	0.006
PLT, ^∗^10^9^/L	205.00 (161.00, 249.25)	207.00 (164.00, 250.00)	196.00 (138.00, 246.50)	0.113
ALT, U/L	33.00 (23.00, 56.00)	32.00 (22.25, 51.75)	56.00 (30.00, 193.00)	<0.001
AST, U/L	72.00 (36.50, 169.5)	67.00 (35.00, 143.00)	225.00 (73.50, 456.00)	<0.001
GGT, U/L	44.00 (27.00, 75.00)	43.00 (27.00, 72.75)	61.00 (29.00, 104.00)	0.007
BUN, mmol/L	6.72 (5.25, 9.37)	6.38 (5.09, 8.50)	10.33 (7.45, 13.15)	<0.001
Creatinine, umol/L	101.00 (82.00, 128.00)	98.00 (81.00, 119.00)	134.00 (109.00, 174.50)	<0.001
Uric acid, umol/L	484.00 (449.00, 542.00)	481.00 (447.00, 535.00)	523.00 (461.00, 637.00)	<0.001
Cystatin C, mg/L	1.22 (0.97, 1.58)	1.17 (0.95, 1.49)	1.65 (1.32, 2.18)	<0.001
CK, U/L	507.00 (186.00, 1368.75)	463.50 (172.00, 1322.50)	745.00 (303.25, 2012.50)	0.002
CKMB, U/L	52.00 (25.00, 127.00)	48.00 (24.00, 117.25)	86.00 (33.00, 190.00)	<0.001
LDH, U/L	375.00 (266.25, 639.75)	350.50 (255.25, 556.75)	695.50 (407.75, 1229.75)	<0.001
*α*-HBDH, U/L	259.00 (173.00, 475.00)	240.00 (165.00, 427.50)	490.50 (273.75, 773.00)	<0.001
CTnT, ng/L	1014.00 (213.50, 3480.00)	786.95 (185.97, 3069.00)	3077.00 (1133.00, 6711.00)	<0.001
BNP, pg/mL	1022.50 (255.15, 3860.75)	884.90 (204.85, 2713.00)	5349.00 (2058.00, 15267.00)	<0.001
Glucose, mmol/L	6.66 (5.56, 8.66)	6.52 (5.44, 8.19)	8.47 (6.41, 11.60)	<0.001
Myoglobin, ng/mL	341.10 (104.50, 910.40)	308.95 (95.96, 820.28)	615.00 (203.50, 2251.00)	<0.001
Diseased vessel identified during procedure				
LM, *n* (%)	13 (2)	13 (2)	0 (0)	0.233
LAD, *n* (%)	213 (33)	185 (33)	28 (31)	0.836
LCX, *n* (%)	70 (11)	62 (11)	8 (9)	0.674
RCA, *n* (%)	157 (24)	134 (24)	23 (26)	0.819
Risk assessment				
GRACE, score	125.00 (102.00, 154.00)	121.00 (101.00, 146.00)	178.00 (140.00, 206.50)	<0.001

Values are expressed as medians with interquartile ranges for continuous data. Other values are presented as numbers and percentages. Shock index: ratio of HR to SBP; SIRI: systemic inflammatory response index; SII: systemic inflammatory reaction index; PLR: ratio of platelets to lymphocytes; NLR: the ratio of neutrophils to lymphocytes; MLR: ratio of monocytes to lymphocytes; OHCA: out-of-hospital cardiac arrest; GRACE: Global Registry of Acute Coronary Events score; *α*-HBDH: *α*-hydroxybutyrate dehydrogenase; BNP: B-type natriuretic peptides.

The article "Clinical Feature-Based Machine Learning Model for 1-Year Mortality Risk Prediction of ST-Segment Elevation Myocardial Infarction in Patients with Hyperuricemia: A Retrospective Study" was published in 2021. Journal: Comput Math Methods Med.

**Table 2:** Comparison of validation results of machine learning models.

Models	Accuracy	AUC	Recall	Precision	F1 value
CatBoost	0.89	0.87	0.33	0.78	0.44
RF	0.89	**0.88**	0.26	**0.82**	0.38
XGBoost	**0.90**	0.83	**0.41**	0.81	**0.51**
LR	0.89	0.82	0.38	0.63	0.46
KNN	0.88	0.75	0.21	0.61	0.31
Model with oversampling (SMOTEENN)					
CatBoost	0.96	0.99	0.98	0.95	0.97
RF	0.95	0.99	0.98	0.94	0.96
XGBoost	0.94	0.98	0.98	0.92	0.95
LR	0.91	0.95	0.92	0.92	0.92
KNN	0.92	0.96	0.98	0.88	0.93
Tradition risk score model					
GRACE score	0.84	0.80	0.46	0.59	0.51

AUC and F1 score: the higher, the better. XGBoost: Extreme Gradient Boosting; RF: random forest; LR: logistic regression; KNN: *K*-nearest neighbors.

**Table 3:** Ensemble of machine learning models.

Ensemble	Accuracy	AUC	Recall	Precision	F1 value
RF+CatBoost+XGBoost	0.90	0.87	0.36	0.72	0.47
XGBoost+LR+KNN	0.90	0.84	0.33	0.72	0.43
RF+LR+KNN	0.89	0.86	0.30	0.71	0.39
RF+XGBoost+LR+KNN	0.90	0.86	0.37	0.73	0.46
All	0.90	0.86	0.37	0.73	0.47

## Data Availability

The datasets are available from the corresponding author upon reasonable request.
